The article "A natural food sweetener with anti-pancreatic cancer properties" was retracted in 2023. Reasons: duplicated images; signs of a paper mill; lack of ethics approval or compliance.

# A natural food sweetener with anti-pancreatic cancer properties

**DOI:** 10.1038/oncsis.2016.28

**Published:** 2016-04-11

**Authors:** C Liu, L-H Dai, D-Q Dou, L-Q Ma, Y-X Sun

**Affiliations:** 1 Key Laboratory of Urban Agriculture (North) of Ministry of Agriculture, Beijing University of Agriculture, Beijing, China; 2 National Engineering Laboratory for Industrial Enzymes, Tianjin Institute of Industrial Biotechnology, Chinese Academy of Sciences, Tianjin, China

## Abstract

Mogroside V is a triterpenoid isolated from the traditional Chinese medical plant *Siraitia grosvenorii*. Mogroside V has a high degree of sweetness and a low calorific content. Herein, we found that mogroside V possesses tumor growth inhibitory activity in *in vitro* and *in vivo* models of pancreatic cancer by promoting apoptosis and cell cycle arrest of pancreatic cancer cells (PANC-1 cells), which may in part be mediated through regulating the STAT3 signaling pathway. These results were confirmed *in vivo* in a mouse xenograft model of pancreatic cancer. In xenograft tumors, Ki-67 and PCNA, the most commonly used markers of tumor cell proliferation, were downregulated after intravenous administration of mogroside V. Terminal deoxynucleotidyl transferase dUTP nick end labeling assays showed that mogroside V treatment promoted apoptosis of pancreatic cancer cells in the xenograft tumors. Furthermore, we found that mogroside V treatment significantly reduced the expression of CD31-labeled blood vessels and of the pro-angiogenic factor vascular endothelial growth factor in the xenografts, indicating that mogroside V might limit the growth of pancreatic tumors by inhibiting angiogenesis and reducing vascular density. These results therefore demonstrate that the natural, sweet-tasting compound mogroside V can inhibit proliferation and survival of pancreatic cancer cells via targeting multiple biological targets.

## Introduction

Cancer poses an important threat to human health, and seriously affects the quality of life. For example, patients with cancer experience fatigue, weakness and high levels of pain. In addition, chemotherapy drugs used in the treatment of cancers have numerous side effects that also seriously affect the quality of life. Therefore, it is particularly important to increase the efficacy of cancer drugs and reduce the side effects of chemotherapy to ensure a sustainable and effective chemotherapy course.

Chemotherapy is one of the most important antitumor therapies. Chemotherapeutic drugs can greatly improve the quality of life and prolong survival, and thus the search for high efficiency chemotherapy drugs with low toxicity is a major focus of oncology research. Although the screening of pharmacologically active compounds in plants is an important approach for developing new drugs, plants that may contain pharmacologically active compounds are widely distributed and numerous, and the compounds are complex. Hence, random screening of plant-derived drugs is laborious. Traditional Chinese medicine uses plants that are proven to be clinically effective for thousands of years, thereby providing a large resource for drug development.^1, 2^ Therefore, screening single compounds that have particularly high efficacy in Chinese herbal medicines may be an important approach for developing new therapies.

Among the plants commonly used in traditional Chinese medicine is *Siraitia grosvenorii*, an endemic plant in China that is mainly grown in Guangxi province, which accounts for more than 90% of the global *S. grosvenorii* production. In 1997, the Chinese Ministry of Health approved *S*. *grosvenorii* saponins as a sweetener in various types of foods. *S*. *grosvenorii* saponins are the main sweetening compounds in *S*. *grosvenorii* and are several hundredfold sweeter than sucrose.

*S*. *grosvenorii* is among the first group of 'Medicinal and Edible' drugs included in the Pharmacopoeia of the People's Republic of China,^3^ which lists the main effects of *S*. *grosvenorii* as 'heat-releasing and lung-moistening, beneficial to the pharynx and voice, facilitating to bowel movement and acting as a laxative.' Currently, studies on *S*. *grosvenorii* are focused on its antioxidant,^4, 5^ anti-inflammatory^6^ and blood lipid- and sugar-reducing potential.^7^ However, thus far, the numerous studies on *S*. *grosvenorii* have not been sufficiently comprehensive. Notably, they have failed to provide a clear mechanism of action and to characterize the full pharmacological effects of this medicinal plant. In particular, the use of *S*. *grosvenorii* in the development of anti-pancreatic cancer drugs has not been explored.

Pancreatic cancer is a malignant disease that affects glucose metabolism.^8, 9^ Thus, pancreatic cancer patients should avoid excessive sugar intake, as chronic excessive consumption of sugar increases the risk of pancreatic cancer. However, most people consume sweet foods and drinks in everyday life. Thus, a means to provide anticancer treatment along with a clinically approved sweetener would be particularly beneficial for pancreatic cancer patients. Herein, it was observed that mogroside V extracted from *S*. *grosvenorii* inhibited pancreatic cancer cell proliferation and survival through the STAT3 pathway both *in vivo* and *in vitro*. These results indicate that mogroside V may be a promising anticancer drug for daily use with relatively few side effects.

## Results

### Mogroside V inhibited the proliferation and survival of PANC-1 cells

We examined the effects of mogroside V (Figure 1a) on the proliferation of PANC-1 cells and other tumor types in liquid cell culture using the MTT assay. As shown in Figure 1b, mogroside V inhibited the proliferation of pancreatic cancer cells and other tumor cell types in a dose- and time-dependent manner, and showed very little cytotoxicity against the non-tumorigenic epithelial cell line L02. To further determine whether the anti-proliferative effects of mogroside V were related to the induction of apoptosis and/or necrosis, mogroside V-treated cells were analyzed with terminal deoxynucleotidyl transferase dUTP nick end labeling (TUNEL) assays. After 24 h of treatment with mogroside V, the percentage of TUNEL-positive cells was increased in a concentration-dependent manner, ranging from 2.91% in the non-treated control cells to 92.25% in the cells treated with 250 μmol/l of mogroside V (Figure 1c).

### Mogroside V induced apoptosis of PANC-1 cells and caused cell cycle arrest at the G0/G1 phase

To further investigate the inhibition of cell proliferation and viability by mogroside V, apoptosis and the cell cycle distribution of PANC-1 cells treated with mogroside V concentrations ranging from 0 to 250 μmol/l were examined using flow cytometry. Annexin V flow cytometry assays revealed that mogroside V caused apoptosis in PANC-1 cells. As illustrated in Figures 2a and b, mogroside V induced apoptosis in PANC-1 cells in a concentration- and time-dependent manner. We further found that z-VAD-fmk, a general caspase inhibitor, inhibited apoptosis of PANC-1 cells induced by treatment with mogroside V for 48 h (Figure 2c). Furthermore, a mogroside V concentration-dependent increase in the G0/G1 ratio was observed, reaching a 1.7-fold increase after exposure to the highest dose (250 μmol/l) compared with that in the untreated cells (Figure 2d).

### Mogroside V altered the level of STAT3 signaling activity

The STAT3 pathway has an important role in cell growth, proliferation and survival, and is implicated in several types of human cancer.^10, 11^ We therefore assessed the effect of mogroside V treatment on this signaling pathway in PANC-1 cells by western blot assays. We found that the level of phosphorylated STAT3 (p-STAT3) in PANC-1 cells was reduced after treatment with mogroside V for 24 h (Figure 3). We further examined whether mogroside V modulated the expression of proteins involved in cell cycle regulation and apoptotic pathways that are downstream of the STAT3 pathway. The expression of the cyclin kinase inhibitors CDKN1A (p21^WAF1^) and CDKN1B (p27),^12, 13, 14^ which are associated with cell cycle arrest in the G0-G1 phase,^15^ was increased by mogroside V in a dose-dependent manner after 24 h. In contrast, the expression of the pro-proliferative cell cycle regulators CCND1 (cyclin D1), CCNE1 (cyclin E1) and CDK2 was decreased after mogroside V treatment.^16^ Furthermore, the expression of the anti-apoptotic proteins BCL2L1 and BCL2 was decreased, whereas that of the proapoptotic CASP3 and BAX proteins was increased after the 24-h mogroside V treatment. In addition, mogroside V suppressed phosphorylation of the kinases upstream of STAT3, including that of JAK2 and TYK2 (Figures 3c and d).

### Evaluation of the antitumor activity of mogroside V *in vivo*

To determine the ability of mogroside V to inhibit tumor growth *in vivo*, we evaluated the antitumor activity of mogroside V against PANC-1 tumors in a nude mouse xenograft model by intravenously injecting experimental mice with different doses of mogroside V 3 days/week for 5 weeks. Tumor growth was significantly inhibited in the mice treated with mogroside V at all doses evaluated compared with that in the control mice (Figure 4a). The mice were killed and the tumors were anatomized 35 days after xenografting. The mean tumor volume in the control mice was 278.6±0.03 mm^3^ compared with 56.4±0.11 mm^3^ in the high-dose mogroside V-treated mice (79.7% decrease; *P*<0.001). The overall tumor weight in the control group was 32.2±1.4 g, whereas it was only 9.2±1.8 g in the mice that had received the high-dose mogroside V treatment (71.4% decrease; Figure 4b). Overall survival rates were estimated by the Kaplan–Meier method, confirming the association between mogroside V treatment and survival (see Figures 4c for the survival curve). Our data demonstrated that mogroside V could not only increase survival of the mice used for the *in vivo* pancreatic cancer model but also that of the mice used for the *in vivo* colon cancer HT29 and laryngeal cancer HEP-2 xenograft models (Supplementary Figure S1). The results of these xenograft experiments were consistent with the in *vitro* data shown in Figure 1b, and indicated that mogroside V might be a potent tumor growth inhibitor.

### Immunohistochemistry analysis (IHC) of tumor cell proliferation, apoptosis and angiogenesis

The potential mechanisms underlying tumor growth inhibition by mogroside V *in vivo* were assessed with IHC assays detecting cell death, cell proliferation and angiogenesis. TUNEL staining of tissue sections (Figure 5) revealed that more cells were TUNEL-positive in the low-dose (57.8% TUNEL-positive), moderate dose (73.1% TUNEL-positive) and high-dose (82.1% TUNEL-positive) mogroside V groups compared with cells in the control group (5.2% TUNEL-positive), indicating that mogroside V induced a high rate of apoptosis in PANC-1 tumor cells.

We next assessed cell proliferation in the tumors using IHC to detect PCNA and Ki-67. The number of cells expressing these markers was significantly decreased in all mogroside V treatment groups compared with that in the control groups (*P*<0.001) (Figure 6). *PCNA* and *Ki-67* mRNA expression *in vivo* was evaluated by real-time–PCR (RT–PCR) assays (Figure 6). Mogroside V clearly reduced *PCNA* and *Ki-67* mRNA expression, which was in accordance with the IHC data shown in Figure 6 (*P*<0.001). Taken together, these data indicated that mogroside V inhibited tumor cell survival and proliferation.

Finally, we determined whether mogroside V affected microvascular density (MVD) and angiogenesis in tumors. As shown in Figure 7a, expression of the pro-angiogenic factor vascular endothelial growth factor (VEGF) was lower in the mogroside V treatment groups (22.82% of the cells was VEGF+ in the highest dosage group) than that in the control group (64.71% of the cells was positive; *P*<0.001); thus, there were 64.73% fewer VEGF-expressing cells after treatment with the highest dose of mogroside V. To examine the effect of mogroside V treatment on MVD in the tumors, blood vessels were labeled with CD31 (Figure 7b) and MVD was calculated according to Weidner's method. The MVD value (Figure 7c) in the mogroside V-treated group (4.11) was significantly lower than that in the control group (37.23; 88.96% decrease, *P*<0.001). These results showed that mogroside V inhibited tumor angiogenesis in a dose-dependent manner.

## Discussion

In this study, a cellular and molecular approach was used to determine the mechanisms underlying cell division and PANC-1 tumor survival regulation by mogroside V. Our findings clearly demonstrated that mogroside V treatment inhibited tumor cell growth, induced apoptosis and caused tumor regression. Moreover, mogroside V inhibited the proliferation of not only pancreatic cancer cells but also that of U937 and A549 cancer cells. In contrast, mogroside V at equivalent concentrations had a minimal effect on normal human liver cells (L02) (Figure 1b). Taken together, these results suggest that mogroside V may be less toxic to normal cells than to cancer cells.

Heretofore, the biochemical targets of mogroside V had not been elucidated. Herein, using western blotting, we demonstrated that mogroside V regulated the protein expression of STAT3. Moreover, mogroside V inhibited the downstream targets of the STAT3 pathway that promote cell proliferation (CCND1, CCNE1 and CDK2), while also upregulating cell cycle inhibitors (CDKN1A and CDKN1B). These effects are in accordance with our finding of a dose-dependent G0-G1 cell cycle arrest in mogroside V-treated PANC-1 cells.^17^ We further found that mogroside V treatment inhibited anti-apoptotic signals downstream of STAT3 (for example, BCL2 and BCL2L1),^18, 19^ which coincided with an increase in the expression of the proapoptotic proteins CASP3 and BAX.^20, 21^ We further found that apoptosis of PANC-1 cells was partially blocked by the caspase inhibitor z-VAD-fmk (Figure 2c), suggesting that mogroside V-induced apoptosis may in part be mediated through the caspase pathway.

Our results obtained using the PANC-1 xenograft models indicated that mogroside V potently inhibited tumor growth *in vivo*. Furthermore, similar to our *in vitro* findings, mogroside V also reduced cell viability and proliferation *in vivo* and reduced p-STAT3 in PANC-1 tumors in a dose-dependent manner (Supplementary Figure S2). TUNEL assays revealed that mogroside V strongly induced apoptosis. Proliferative activity in xenograft tumors was assessed by IHC for Ki-67 and PCNA. Ki-67 is a cell proliferation marker that is expressed in all phases of the cell cycle, except the G0 phase.^22, 23^ PCNA, a 36-kD DNA polymerase delta auxiliary protein involved in the proliferation of neoplastic and non-neoplastic cells,^24, 25^ is specifically expressed in proliferating cell nuclei and is commonly used to measure tumor cell proliferation. The expression of both Ki-67 and PCNA was reduced in PANC-1 xenograft tumors in all mogroside V treatment groups compared with that in the control groups and corresponded with reductions in tumor weight. Thus, mogroside V may act pharmacologically by inhibiting the proliferation of PANC-1 cells, while also inducing apoptosis, thereby subsequently limiting pancreatic tumor growth.

Finally, we found that VEGF expression and MVD were diminished in PANC-1 xenograft tumors. VEGF has an important role in angiogenesis in both tumors and healthy tissues.^26, 27^ These data thus suggest that mogroside V may prevent pancreatic tumor growth by inhibiting angiogenesis through a VEGF-dependent mechanism. Consequently, this would lead to decreased MVD and, hence, diminished tumor growth. STAT3 is an essential mediator of VEGF transcription by directly binding to the VEGF promoter, thereby inducing angiogenesis.^28, 29^ Our study showed that mogroside V significantly inhibited the activation of STAT3 protein in PANC-1 cancer cells concomitantly with reducing VEGF protein levels *in vivo*. This finding suggests that the anti-angiogenic effects of mogroside V may be due to the ability of mogroside V to prevent STAT3 activation.

Our study was limited by the fact that we did not explore the effects of a stable overexpression of STAT3 or deletion of STAT3 in the PANC-1 cells used as tumor xenografts. The efficacy of mogroside V treatment under these conditions is not known and will be the focus of our future studies.

In conclusion, we have found through *in vitro* and *in vivo* experiments that mogroside V inhibited pancreatic cancer cell proliferation and promoted tumor apoptosis. Moreover, mogroside V interfered with angiogenesis in pancreatic tumors. Therefore, our results suggest that mogroside V may be a potential anticancer compound that acts on the STAT3 pathway. Moreover, we demonstrated that mogroside V could not only prevent tumor progression *in vivo* but also increase survival of the mice, indicating that this natural compound might possess potential therapeutic activity. Given that mogroside V is a natural sweetener that has been approved by the United States Food and Drug Administration, it may be used for daily consumption as an additive in foods and drinks to prevent or treat pancreatic cancer.

## Materials and methods

### Drugs and reagents

Mogroside V was purchased from Sigma-Aldrich (St Louis, MO, USA). All other reagents were also purchased from Sigma-Aldrich unless specified otherwise.

### Cell lines and cell culture

The human pancreatic adenocarcinoma cell line PANC-1 was obtained from Shanghai Cell Biology Institute (Shanghai, China). PANC-1 cells were cultured in Dulbecco's modified Eagle's medium supplemented with 10% heat-inactivated fetal bovine serum (Gibco, Grand Island, NY, USA), 100 μg/ml streptomycin and 100 U/ml penicillin under a humidified 5% CO_2_ atmosphere at 37 °C. Human pancreatic adenocarcinoma cell lines MiaPaCa-2 and CFPAC-1, A549 lung adenocarcinoma, human U937 and L02 normal human liver cells were obtained from Shanghai Cell Biology Institute. MiaPaCa-2 and CFPAC-1 cells were cultured in Dulbecco's modified Eagle's medium and A549, U937 and L02 cells were cultured in RPMI1640. All media were supplemented with heat-inactivated fetal bovine serum (10%), 100 μg/ml streptomycin and 100 U/ml penicillin. The cells were maintained at 37 °C with 5% CO_2_.

### *In vitro* cellular proliferation (MTT) and TUNEL assays

Cells were added to 96-well cell culture plates at an initial concentration of 1 × 10^4^ cells/ml and were incubated with the indicated concentrations of mogroside V. After 24 or 72 h of incubation, MTT solution (5 mg/ml) was added to the wells and the cells were incubated for another 4 h. The growth medium was removed and formazan crystals formed by oxidation of the MTT dye were analyzed by measuring the absorbance at 490 nm using an ELISA reader.^30, 31^

Cells were labeled for apoptotic DNA strand breaks by a TUNEL reaction using the *In Situ* Cell Death Detection Kit (POD; Roche Applied Science, Indianapolis, IN, USA) to determine the percentage of cells undergoing mogroside V-induced apoptosis, and were incubated with antidigoxigenin peroxidase for 30 min using DAB substrate. The apoptotic cells were visualized using light microscopy (Olympus, Tokyo, Japan). For quantifying apoptotic cells, the percentage of TUNEL-positive cells in a cancer cell population of 300 cells was determined in five random fields per glass slide.

### Cell cycle analysis and measurement of apoptosis

Cell cycle status was determined using flow cytometry. PANC-1 cells were analyzed for alterations in their cell cycle after treatment with mogroside V for 24 h. The cells used for the flow cytometry experiments were both floating and adherent cells. After the cells were fixed with 70% methanol, they were treated with RNase A and were exposed to propidium iodide for flow cytometry analysis. Detection of apoptosis was performed using Annexin V-FITC staining with an Annexin V assay kit (Annexin V-FITC Apoptosis Detection Kit; BD Pharmingen, San Diego, CA, USA). Briefly, PANC-1 cells (1 × 10^5^ cells) were cultured with mogroside V for 24 to 96 h, followed by labeling with Annexin V-FITC and propidium iodide according to the manufacturer's instructions. The percentage of cells undergoing apoptosis in the control and mogroside V-treated cells was analyzed using flow cytometry. In the apoptosis inhibition assays, cells were incubated with or without mogroside V for 48 h in the presence or absence of the apoptosis inhibitor zVAD (20 μmol/l). The results were evaluated with the CellQuest software (BD Biosciences, San Jose, CA, USA).

### Western blot assay

Cells were treated with mogroside V for 24 h and were lysed at 4 °C in lysis buffer (0.05 M Tris-HCl, pH 7.4, 1% Triton X-100, 0.1 M NaCl, 1% sodium deoxycholate and 0.1% SDS) containing 1 mM phenylmethanesulfonyl fluoride and a protease inhibitor. The insoluble protein lysate was removed by centrifugation. About 15 μg of protein from the cell lysates were separated by 12% SDS–PAGE and were subsequently transferred onto a polyvinylidene fluoride membrane. The following primary antibodies were used for western blot analysis: STAT3 (1:1000 dilution), phospho-(p)-STAT3, CDKN1A, CDKN1B (p27), BCL2 and β-actin (all from Sigma-Aldrich). After incubation with the appropriate secondary antibodies (all from Sigma-Aldrich), the membranes were developed with ECL plus (ECL, Amersham Biosciences, GE Healthcare, Pittsburgh, PA, USA). Densitometric measurements of the protein bands were performed using the GS-800 imaging densitometer (Bio-Rad, Hercules, CA, USA).

### PANC-1 xenograft model and tumor treatment

The *in vivo* characteristics of the pancreatic tumors were investigated in a BALB/c nude mice xenograft model. Approximately 8-week-old male nude BALB/c mice from Vital River (Charles River Ltd. Co., Beijing, China) were maintained in a pathogen-free environment. To establish a xenograft tumor model, PANC-1 cells (1 × 10^7^) were injected subcutaneously in the flank of the mice. The mice were randomly divided into the following five groups: (i) untreated control group, (ii) NC group (normal saline), (iii) 2 mg/kg b.w. mogroside V group, (iv) 10 mg/kg b.w. mogroside V group and (v) 30 mg/kg b.w. mogroside V. Mogroside V was dissolved in normal saline and was administered to the mice in a volume of 0.1 ml. The tumors were measured with a vernier caliper every 3 days. The tumor volumes were determined by measuring the length (l) and width (w) of the tumors, and by calculating the tumor volume (V=*w*^*2*^*l*/2).^32^ After 5 weeks, the mice were killed and the tumors were dissected and weighed. The inhibition rate of tumor growth was calculated using the following formula: tumor growth inhibition rate (%)=(1−M_T_/M_C_) × 100, where M_T_ and M_C_ are the mean tumor masses of the treatment and control groups, respectively. Animal use complied with Beijing University of Agriculture Animal Welfare Guidelines.

### Immunohistochemistry

Following dissection, the tumor tissues were fixed immediately in 10% phosphate-buffered formalin and were embedded in paraffin. Proliferation of pancreatic cancer cells was estimated by IHC staining with either a mouse monoclonal PCNA or Ki-67 antibody (Santa Cruz Biotechnology, Inc., Santa Cruz, CA, USA), and the number of PCNA- and Ki-67-positive cells in a population of 200 cells sampled at × 400 magnification was counted. The proliferating cell nuclear antigen labeling index and Ki-67 labeling index were subsequently calculated. After treatment with mogroside V, vascularization was evaluated in CD31- and VEGF-immunostained tissue sections. The MVD was calculated according to Weidner's method.^33, 34^ TUNEL immunohistochemistry was performed using an *In Situ* Cell Death Detection Kit (Roche Diagnostics GmbH, Mannheim, Germany) according to the manufacturer's instructions.

### Quantitative real-time PCR (RT–PCR) analysis

The expression levels of the mRNA transcripts of interest were determined by RT–PCR assays.^35^ Total RNA was isolated from fresh tumor tissues with TRIzol Reagent (Invitrogen, Carlsbad, CA, USA). Oligo(dT)-primed RNA (2 μg) was reverse-transcribed with SuperScript II reverse transcriptase (Promega, Madison, WI, USA) according to the manufacturer's instructions. The obtained cDNA was used to determine the mRNA amount of *PCNA* and *Ki-67* by PCR with Taq DNA polymerase (Fermentas, Thermo Fisher Scientific, Inc., Waltham, MA, USA). *GAPDH* was used as an internal control. The following primer sequences were used for amplification of *PCNA, Ki-67* and *GAPDH*: *PCNA* forward 5′-CCTGCTGGGATATTAGCTCCA-3′ and reverse 5′-CAGCGGTAGGTGTCGAAGC-3′ (Tm=60 °C, 109 bp); *Ki-67* forward 5′-GCCTGCTCGACCCTACAGA-3′ and reverse 5′-GCTTGTCAACTGCGGTTGC-3′ (Tm=60 °C, 127 bp); *GAPDH* forward 5′-CTGGGCTACACTGAGCACC-3′ and reverse 5′-AAGTGGTCGTTGAGGGCAATG-3′ (Tm=60 °C, 101 bp). The resultant PCR samples were analyzed by gel electrophoresis (1.5% agarose). The DNA bands were examined using a Gel Documentation System (Model Gel Doc 2000; Bio-Rad, Hercules, CA, USA).

### Statistics

The data were presented as the means±s.d. of three independent experiments for the *in vitro* study and *n*=6 for the *in* *vivo* study. Statistical significance was determined using Student's *t*-test. Survival was estimated using the Kaplan–Meier method and the values obtained were compared using the log-rank test. Statistical analysis was performed using GraphPad Prism 5 (GraphPad Software, Inc., La Jolla, CA, USA) with *P*<0.05 considered statistically significant

## Figures and Tables

**Figure 1:** Mogroside V inhibits the proliferation and induces apoptosis in cultured cells. (**a**) Chemical structure of mogroside V extracted from *S. grosvenorii.* (**b**) Graph of MTT assay results indicating the rate of cell proliferation inhibition in PANC-1 and other tumor cell types treated with mogroside V. (**c**) Representative images of cells plated onto slides for TUNEL reaction apoptosis assays. The percentage of cells undergoing apoptosis increased with increasing mogroside V concentrations. The results were obtained in three independent experiments.

**Figure 2:** Apoptosis and cell cycle analysis of PANC-1 cells treated with mogroside V. (**a**) Representative flow cytometry plots from Annexin V assays indicating that mogroside V induced apoptosis in PANC-1 cells in a concentration-dependent manner and (**b**) a time-dependent manner. (**c**) PANC-1 cells were treated with or without mogroside V (20 μmol/l) for 48 h in the presence or absence of the apoptosis inhibitor zVAD (20 μmol/l). (**d**) Graphic indicating the cell cycle stages that were analyzed using flow cytometry. The percentage of cells in the G0/G1, S or G2/M phase of the cell cycle is indicated. An increase in the G0-G1 population was observed in the mogroside V-treated cells. The results were obtained in three independent experiments.

**Figure 3:** The effect of mogroside V on the STAT3 pathway. PANC-1 cells were exposed to various concentrations of mogroside V for 24 h and the target proteins were detected by immunoblotting using specific antibodies. (**a**) Phosphorylation of STAT3 (p-STAT3) and the expression of proteins downstream of the STAT3 pathway were suppressed in the mogroside V-treated cells. (**b**) A tentative depiction of the regulation of the STAT3 signaling pathway in PANC-1 cells by mogroside V. (**c**) The phosphorylation of STAT3 to p-STAT3 and protein expression of STAT3, P-JAk2, JAK2, P-TYK2 and TYK2 in mogroside V-treated PANC-1 cells and MiaPaCa-2 cells (**d**) were examined using western blotting. Beta-actin expression served as a loading control. The results were obtained in three independent experiments.

**Figure 4:** Mogroside V inhibits PANC-1 cell tumor growth in a mouse xenograft tumor model. Mice were implanted with PANC-1 cells and were randomly divided into five groups: a Control group, NC (normal saline) and three treatment groups receiving doses of 2, 10 or 30 mg/kg b.w. mogroside V three times a week. (**a**) The average volume of the tumor xenografts in the five groups, as measured with vernier calipers after the mice were killed and the tumor was anatomized 35 days post treatment. (**b**) The average weight of the tumor xenografts in the five groups. The tumor weight was significantly lower in the mogroside V treatment groups than that in the control and NC groups. For statistical analysis, mogroside V-treated mice were compared with vehicle control mice using Student's *t*-tests; **P<0.01 and ***P<0.001 versus the control values. (**c**) Kaplan–Meier survival analysis showed that mogroside V treatment was significantly correlated with overall survival (*P*<0.01, using log-rank test, *P*<0.05 was considered significant).

**Figure 5:** Immunohistochemical analysis of PANC-1 cell xenograft tumor apoptosis. Cells were stained using the TUNEL method and were scored for apoptosis by comparison with the vehicle control. The images on the left illustrate the level of TUNEL staining in the PANC-1 cells comprising the tumor in the control and mogroside V treatment groups. The graphs on the right indicate a mogroside V concentration-dependent increase in TUNEL staining as determined by counting tissue sections from eight independent tumors. For statistical analysis, mogroside V-treated mice were compared with vehicle control mice using Student's *t*-tests; ***P<0.001 versus the control values.

**Figure 6:** The effect of mogroside V on the expression of PCNA and Ki-67 in PANC-1 xenograft tumors. (**a**) Images of immunohistochemical staining and RT–PCR analysis indicating that mogroside V inhibits PCNA expression. (**b**) Images of immunohistochemical staining and RT–PCR analysis indicating that mogroside V inhibited PCNA expression. The data represent the means±s.d. Statistical analysis was performed using the Student's *t*-test; ***P<0.001 versus the control values.

**Figure 7:** Determination of angiogenesis by immunohistochemical analysis of VEGF and CD31 expression. VEGF and CD31 protein expression was significantly downregulated in PANC-1 tumors. (**a**) Immunohistochemical staining of VEGF in xenograft tumors of each of the indicated control and mogroside V treatment groups. (**b**) Representative images of CD31 immunohistochemical staining in xenograft tumors of each of the indicated control and mogroside V treatment groups. (**c**) Graph of the MVD measurements in sections of xenograft tumors as determined by CD31 expression. The data represent the means±s.d. Statistical analysis was performed using the Student's *t*-test. *P<0.05, **P<0.01 and ***P<0.001 versus the control values.

## References

[bib1] Efferth T, Li PC, Konkimalla VS, Kaina B. From traditional Chinese medicine to rational cancer therapy. Trends Mol Med 2007; 13: 353–361.1764443110.1016/j.molmed.2007.07.001

[bib2] Parekh HS, Liu G, Wei MQ. A new dawn for the use of traditional Chinese medicine in cancer therapy. Mol Cancer 2009; 8: 21.1929867710.1186/1476-4598-8-21PMC2664781

[bib3] Commission C: Pharmacopoeia of the People's Republic of China. China Medical Science Press: Beijing, China, 2010, pp 197.

[bib4] Chen W, Wang J, Qi X, Xie B. The antioxidant activities of natural sweeteners, mogrosides, from fruits of Siraitia grosvenori. Int J Food Sci Nutr 2007; 58: 548–556.1785249610.1080/09637480701336360

[bib5] Qi X, Chen W, Zhang L, Shan X, Song Y. Study on the inhibitory effects of natural sweetner mogrosides on radical and lipid peroxidation. Scientia Agricultura Sinica 2006; 39: 382–388.

[bib6] Di R, Huang M-T, Ho C-T. Anti-inflammatory activities of mogrosides from Momordica grosvenori in murine macrophages and a murine ear edema model. J Agric Food Chem 2011; 59: 7474–7481.2163111210.1021/jf201207m

[bib7] Qi X-Y, Chen W-J, Zhang L-Q, Xie B-J. Mogrosides extract from Siraitia grosvenori scavenges free radicals *in vitro* and lowers oxidative stress, serum glucose, and lipid levels in alloxan-induced diabetic mice. Nutr Res 2008; 28: 278–284.1908342010.1016/j.nutres.2008.02.008

[bib8] Gapstur SM, Gann PH, Lowe W, Liu K, Colangelo L, Dyer A. Abnormal glucose metabolism and pancreatic cancer mortality. JAMA 2000; 283: 2552–2558.1081511910.1001/jama.283.19.2552

[bib9] Permert J, Ihse I, Jorfeldt L, Von Schenck H, Arnqvist H, Larsson J. Pancreatic cancer is associated with impaired glucose metabolism. Acta Chirurgica 1993; 159: 101–107.8098623

[bib10] Bromberg JF, Wrzeszczynska MH, Devgan G, Zhao Y, Pestell RG, Albanese C et al. Stat3 as an oncogene. Cell 1999; 98: 295–303.1045860510.1016/s0092-8674(00)81959-5

[bib11] Darnell JE. Validating Stat3 in cancer therapy. Nat Med 2005; 11: 595–596.1593746610.1038/nm0605-595

[bib12] Soos TJ, Kiyokawa H, Yan JS, Rubin MS, DeBlasio A, Giordano A et al. Formation of p27-CDK complexes during the human mitotic cell cycle. Cell Growth Differ 1996; 7: 135–146.8822197

[bib13] Nakayama K, Nagahama H, Minamishima YA, Miyake S, Ishida N, Hatakeyama S et al. Skp2-mediated degradation of p27 regulates progression into mitosis. Dev Cell 2004; 6: 661–672.1513049110.1016/s1534-5807(04)00131-5

[bib14] Harper JW, Adami GR, Wei N, Keyomarsi K, Elledge SJ. The p21 Cdk-interacting protein Cip1 is a potent inhibitor of G1 cyclin-dependent kinases. Cell 1993; 75: 805–816.824275110.1016/0092-8674(93)90499-g

[bib15] Ma X, Wang S, Du R, Ye Y, Yan F, Cui Z. Stat3 signal transduction pathway orchestrates G1 to S cell cycle transition in colon cancer cells. Beijing Da Xue Xue Bao 2003; 35: 50–53.12920809

[bib16] Toyoshima H, Hunter T. p27, a novel inhibitor of G1 cyclin-Cdk protein kinase activity, is related to p21. Cell 1994; 78: 67–74.803321310.1016/0092-8674(94)90573-8

[bib17] McClure C, Ali E, Youssef D, Yao ZQ, McCall CE, El Gazzar M. NFI-A disrupts myeloid cell differentiation and maturation in septic mice. J Leukoc Biol 2016; 99: 201–211.2625991410.1189/jlb.4A0415-171RRPMC4673479

[bib18] Zhou Y, Li M, Wei Y, Feng D, Peng C, Weng H et al. Down-regulation of GRIM-19 expression is associated with hyperactivation of STAT3-induced gene expression and tumor growth in human cervical cancers. J Interferon Cytokine Res 2009; 29: 695–704.1964290610.1089/jir.2009.0003PMC2988461

[bib19] Koskela HL, Eldfors S, Ellonen P, van Adrichem AJ, Kuusanmäki H, Andersson EI et al. Somatic STAT3 mutations in large granular lymphocytic leukemia. N Engl J Med 2012; 366: 1905–1913.2259129610.1056/NEJMoa1114885PMC3693860

[bib20] Wang X, Liu B, Qu B, Xing H, Gao S, Yin J et al. Silencing STAT3 may inhibit cell growth through regulating signaling pathway, telomerase, cell cycle, apoptosis and angiogenesis in hepatocellular carcinoma: potential uses for gene therapy. Neoplasma 2010; 58: 158–171.10.4149/neo_2011_02_15821275467

[bib21] Nielsen M, Kaestel C, Eriksen K, Woetmann A, Stokkedal T, Kaltoft K et al. Inhibition of constitutively activated Stat3 correlates with altered Bcl-2/Bax expression and induction of apoptosis in mycosis fungoides tumor cells. Leukemia 1999; 13: 735–738.1037487810.1038/sj.leu.2401415

[bib22] Scholzen T, Gerdes J. The Ki-67 protein: from the known and the unknown. J Cell Physiol 2000; 182: 311–322.1065359710.1002/(SICI)1097-4652(200003)182:3<311::AID-JCP1>3.0.CO;2-9

[bib23] Gerdes J, Lemke H, Baisch H, Wacker H-H, Schwab U, Stein H. Cell cycle analysis of a cell proliferation-associated human nuclear antigen defined by the monoclonal antibody Ki-67. J Immunol 1984; 133: 1710–1715.6206131

[bib24] Kelman Z. PCNA. structure, functions and interactions. Oncogene 1997; 14: 629–640.903837010.1038/sj.onc.1200886

[bib25] Maga G, Hübscher U. Proliferating cell nuclear antigen (PCNA): a dancer with many partners. J Cell Sci 2003; 116: 3051–3060.1282973510.1242/jcs.00653

[bib26] Neufeld G, Cohen T, Gengrinovitch S, Poltorak Z. Vascular endothelial growth factor (VEGF) and its receptors. FASEB J 1999; 13: 9–22.9872925

[bib27] Holash J, Maisonpierre P, Compton D, Boland P, Alexander C, Zagzag D et al. Vessel cooption, regression, and growth in tumors mediated by angiopoietins and VEGF. Science 1999; 284: 1994–1998.1037311910.1126/science.284.5422.1994

[bib28] Kim BH, Lee Y, Yoo H, Cui M, Lee S, Kim SY et al. Anti-angiogenic activity of thienopyridine derivative LCB03-0110 by targeting VEGFR-2 and JAK/STAT3 Signalling. Exp Dermatol 2015; 24: 503–509.2580846310.1111/exd.12698

[bib29] Yang C, Lee H, Pal S, Jove V, Deng J, Zhang W et al. B cells promote tumor progression via STAT3 regulated-angiogenesis. PLoS ONE 2013; 8: e64159.2373419010.1371/journal.pone.0064159PMC3667024

[bib30] Gerhardt D, Bertola G, Dietrich F, Figueiró F, Zanotto-Filho A, Moreira Fonseca JC et al. Boldine induces cell cycle arrest and apoptosis in T24 human bladder cancer cell line via regulation of ERK, AKT, and GSK-3β. Urol Oncol 2014; 32: 36.e1–36.e9.10.1016/j.urolonc.2013.02.01224239461

[bib31] Adler J, Jarvis K, Marsh K, Klein L, Clement J. Preclinical *in vivo* efficacy of two 9-dihydrotaxane analogues against human and murine tumors. Br J Cancer 1996; 73: 560–565.860508710.1038/bjc.1996.98PMC2074348

[bib32] Carie A, Sebti S. A chemical biology approach identifies a beta-2 adrenergic receptor agonist that causes human tumor regression by blocking the Raf-1/Mek-1/Erk1/2 pathway. Oncogene 2007; 26: 3777–3788.1726002510.1038/sj.onc.1210172

[bib33] Gasparini G, Weidner N, Bevilacqua P, Maluta S, Dalla Palma P, Caffo O et al. Tumor microvessel density, p53 expression, tumor size, and peritumoral lymphatic vessel invasion are relevant prognostic markers in node-negative breast carcinoma. J Clin Oncol 1994; 12: 454–466.750985110.1200/JCO.1994.12.3.454

[bib34] Toi M, Inada K, Suzuki H, Tominaga T. Tumor angiogenesis in breast cancer: its importance as a prognostic indicator and the association with vascular endothelial growth factor expression. Breast Cancer Res Treat 1995; 36: 193–204.853486710.1007/BF00666040

[bib35] Peltier HJ, Latham GJ. Normalization of microRNA expression levels in quantitative RT-PCR assays: identification of suitable reference RNA targets in normal and cancerous human solid tissues. RNA 2008; 14: 844–852.1837578810.1261/rna.939908PMC2327352

